# Efficacy and safety of PARP inhibitors as the maintenance therapy in ovarian cancer: a meta-analysis of nine randomized controlled trials

**DOI:** 10.1042/BSR20192226

**Published:** 2020-03-18

**Authors:** Fengping Shao, Jun Liu, Yaoyun Duan, Li Li, Liqun Liu, Cai Zhang, Shanyang He

**Affiliations:** 1 Department of Obstetrics and Gynecology, The First Affiliated Hospital, Sun Yat-sen University, Zhongshan Second Road 58, Guangzhou 510080, Guangdong, P. R. China; 2 School of Chemical Biology and Biotechnology, State Key Laboratory of Chemical Oncogenomics, Peking University Shenzhen Graduate School, Shenzhen, China, 518055

**Keywords:** Adverse events, BRCA, Efficacy and safety, Ovarian cancer, PARP inhibitors

## Abstract

Purpose: Poly ADP ribose polymerase (PARP) inhibitors can effectively kill cancer cells by restraining the activity of DNA repair enzymes and utilizing the characteristics of BRCA mutations. This article evaluates the efficacy and safety of PARP inhibitors (PARPis) in the maintenance treatment of ovarian cancer.

Method: We searched for clinical trials in electronic databases. PARPis efficacy were evaluated by the hazard ratios (HR) and its 95% confidence intervals (95% CI) of overall survival (OS) and progression-free survival (PFS) between the PARPis groups and placebo groups, while the PARPis’ safety was assessed by relative risk (RR) values of adverse events (AEs) between the two arms.

Results: The immature OS data manifested that patients with BRCA mutation receiving PARPis therapy versus placebo therapy appeared to have longer OS (HR = 0.78, 95%CI = 0.61–1.01; *P* = 0.06). Compared with placebo group, PARP group had a significant advantage in PFS in ovarian cancer patients with BRCA wild-type (BRCAwt), BRCA mutation (BRCAm), BRCA status unclassified, BRCA1 mutation subgroup and the BRCA2 mutation subgroup (BRCAwt: HR = 0.53, 95%CI = 0.42–0.68, *P* < 0.00001; BRCAm: HR = 0.30, 95%CI = 0.26–0.34, *P* < 0.00001; BRCA status unclassified: HR = 0.52, 95%CI = 0.41–0.66, *P* < 0.00001; BRCA1m: HR = 0.38, 95%CI = 0.29–0.48, *P* < 0.00001; BRCA2m: HR = 0.23, 95%CI = 0.10–0.57, *P* = 0.001). Our analysis revealed the incidence rates for AEs of grade ≥3 (grades 3 to 4) and serious AEs in PARPis group were 55.19% and 26.29%, respectively.

Conclusion: Our meta-analysis demonstrates that PARPis therapy can significantly improve PFS in ovarian cancer patients, but it has no benefit in OS. However, the therapy is associated with a significant increase in the risk of AEs of grade ≥ 3 and serious AEs.

## Background

Based on American cancer statistics in 2019, ovarian cancer is the 11th most common cancer, with approximately 22,530 newly diagnosed ovarian cancer cases, and the 5th leading cause of cancer-related death, with estimated 13,980 ovarian cancer deaths [1]. Ovarian cancer patients are characterized by late-stage presentation, easy relapse and metastasis, no chance to radical surgery, which ultimately lead to stagnation of mortality statistics. Ovarian cancer is a diverse and genomic complex disease, which has attracted worldwide attention [2]. Women with inherited mutations in BRCA1 or BRCA2 had an increased risk of ovarian cancer, and for BRCA1 or BRCA2 mutation carriers, the lifetime risk of ovarian cancer were 54% and 23%, respectively [3]. However, compared with mutation-negative patients, patients carrying BRCA mutations have an advantage in progression-free and overall survival, and more frequently respond to both platinum-based chemotherapy and poly (adenosine diphosphate [ADP]–ribose) polymerase (PARP) inhibitors [4,5]. BRCA is known to be involved in homologous recombination [6–8], and the targeted inhibition of specific DNA repair pathways may provide an appropriate treatment for cancer [7]. BRCA-mutation positive epithelial ovarian cancer (EOC) patients appear impaired ability to repair double-stranded DNA breaks via homologous recombination, which may partly explain the molecular basis for heightened sensitivity to platinum and PARPis, as well as better survival compared with nonhereditary EOC patients [4,9–11].

PARPis are a class of molecule-targeting agents suppressing PARP enzymes activity. BRCA1 or BRCA2 dysfunction deeply appears the susceptibility of cancer cells to the inhibition of PARP enzymatic activity, leading to defects in DNA damage repair by homologous recombination, which results in cell death [6,7]. According to our latest search results, nine randomized controlled trials (RCTs) have shown that PARPis have shown impressive results in the treatment of ovarian cancer [10,12–16]. Therefore, this meta-analysis aimed to update and evaluate the efficacy of PARPis in different status of BRCA ovarian cancer, and to assess the safety of them in detail according to the grade and type of AEs.

## Method

### Search strategy

We systematically searched PubMed, Web of Science, Embase, Cochrane CENTRAL and ClinicalTrials.gov from inception to January 2020 for all RCTs. For database search we used “(‘ovarian cancer’ OR ‘ovarian carcinoma’ OR ‘ovarian neoplasm’ OR ‘ovarian tumor’) AND (‘parp’ OR ‘parpi’ OR ‘olaparib’ OR ‘niraparib’ OR ‘rucaparib’) AND (‘randomized’ OR ‘randomised’ OR ‘trial’ OR ‘placebo’)” as the search terms in all fields. Wherever possible, we searched for references to relevant articles to identify potential information that had not already been retrieved. The search was restricted to articles published in English.

### Inclusion criteria

The relevant clinical trials on the efficacy and safety of PARPis therapy were included, if they qualified for a randomized controlled trial with or without blinding. Besides, accepted articles should also meet the following criteria: (1) The trial involved the study of high-grade serous or endometrioid ovarian cancer, primary peritoneal cancer, or fallopian-tube cancer with or without BRCA1 or BRCA2 mutations, platinum-sensitive or platinum-resistant. (2) The trial compared PARPis with other interventions such as placebo or other chemotherapy drugs. (3) The study provided available data to calculate the HR of OS or PFS and RR of AEs.

### Exclusion criteria

Exclusion criteria excluded: (1) The trial was not randomized control trial. (2) Literature reviews, or Case reports, (3) Phase I clinical trial. (4) Duplicate publication. (5) Intervention only included the PARPi (PARPi) group for ovarian cancer. For example, we excluded the articles (Swisher 2017) because they aimed to investigate molecular predictors of rucaparib sensitivity, rather than to evaluate efficacy and safety by comparing it with placebo [17]. Updated and published follow-up data were considered for one trial to analyze.

### Data extraction

Two investigators independently reviewed the whole content of each eligible literature, including supplements, and extracted the data using a pilot-tested data extraction sheet.

The following contents was included in the extraction sheet: first author; year of publication; phase of clinical trial; tumor type and clinical stage; number of patients enrolled; platinum status; BRCA status; interventions; hazard ratios (HR)for OS and PFS and their 95% confidence intervals (CIs); numbers of AEs with different grades and types; and other necessary information.

### Statistical analysis

The data of the analysis were extracted from the selected literature, and all meta-analysis were performed using Review Manager 5.0 (http://www.cochrane.org). Statistical heterogeneity was analyzed using Cochran’s *Q*-test and inconsistency (*I*^2^) statistics; *P* ≤ 0.10 or I2≥50% indicate significant heterogeneity. If there is no heterogeneity, a fixed-effect model (*P* > 0.10 and *I*^2^ < 50%) is used [18], otherwise a random effects model (*P* ≤ 0.10 or *I*^2^ ≥ 50%) is used [19]. HR and 95%CI were used to analyze the OS and PFS between PARPis group and control group. In addition, pooled risk ratio (RR), 95%CI and incidence rate were used to analyze AEs with different degrees via a meta-analysis. For all analyses, *P* < 0.05 was refer to indicate statistical significance.

## Results

### Literature search

A total of 2631 records were identified from all searched databases, and 2321 articles were automatically deleted by selecting the type of articles for clinical trials about human. About 166 articles were retained after excluding duplicates and phase I trial by reading titles and abstracts. After assessing the titles, abstracts and full texts of the article of retained articles, 157 were excluded for the following reasons: reviews; single-arm trials; non-randomized control; non-clinical studies of PFS and OS; non-research ovarian cancer and others do not meet the selection criteria. Finally, 9 randomized controlled trials were included in the final analysis [13,20–28]. The flowchart of the trial selection process is shown in Figure 1.

**Figure 1:** Flow diagram for selection of studies

### Characteristics of the included studies

The characteristics of the nine selected trials are summarized in Table 1. Among nine randomized controlled trials, two were phase II trials, and the other seven were phase III trials, involving 4526 patients in the pooled analyses. In the nine trials included, the therapeutic effects and safety of PARPis including olaparib, rucaparib, veliparid and niraparib as maintenance therapy were evaluated, and that of olaparib were evaluated in five trials. The last four trials including Moore 2018, Coquard 2019, Martin 2019 and Coleman 2019 focused on PARPi as the maintenance therapy for newly diagnosed advanced ovarian cancer, while the earlier five trials including Ledermann 2014, Oza 2014, Mirza 2016, Lauraine 2017 and Coleman 2017 investigated PARPis for recurrent and refractory platinum-sensitive ovarian cancer. When comparing olaparib with placebo in BRCA mutation patients, the HR is gradually reduced with increasing therapeutic doses of olaparib in these studies [13,21,23,24,26], which means a positive dose–response relationship between clinical efficiency and olaparib dosage. In Oza 2014 and Coleman 2019, the intervention regimen of the experimental group was PARPi combined with chemotherapy, followed by PARPi alone for maintenance therapy, while the control group was not further treated in the maintenance phase of the study after chemotherapy. Coquard 2019 reported the efficacy and safety of combination maintenance olaparib and bevacizumab in patients. Although Oza 2014 and Coleman 2019 [13] assessed not only AEs in the treatment phase of PARPi combined with chemotherapy, but also AEs in the maintenance phase of PARPi monotherapy, in this meta-analysis, we only analyzed the AEs at monotherapy maintenance phase. In Miza 2016 [22], ovarian cancer patients with homologous recombination deficiency plus somatic BRCA mutation (HRD positive/sBRCA mutation) and with a germline BRCA mutation (gBRCA mutation) were included in the BRCA mutation group for meta-analysis. In Coleman 2017, ovarian cancer patients with BRCA wild-type were subdivided into high loss of heterozygosity (LOH), indeterminate LOH and low LOH.

**Table 1:** Characteristics of the trials included in the meta-analysis

Trial	Phase	Year	Treatment arms	Therapeutic schedule		Patients (Exp/Con)	Platinum status and clinical stage	BRCA status	Median PFS (BRCA mutation group)
Ledermann 2012,2014,2016	II	2012,2014,2016	Olaparib vs Placebo	Experimental: olaparib 600 mg bid Control: placebo	maintenance monotherapy	136/129	platinum-sensitive recurrent, high grade serous ovarian cancer	BRCA1/2 mutation BRCA wild-type	Experimental:8.3 months Control:4.3 months (HR:0.18, *P* < 0.0001)
Oza 2014	II	2014	Olaparib plus chemotherapy vs Chemotherapy	Experimental: olaparib (200 mg capsules bid) plus chemotherapy, then olaparib monotherapy (400 mg bid) Control: chemotherapy then no further treatment	combination with chemotherapy and maintenance monotherapy	81/81	platinum-sensitive recurrent, high grade serous ovarian cancer	BRCA1/2 mutation BRCA wild-type BRCA not available	Experimental: not reported Control:9.7 months (HR:0.21, *P* < 0.0015)
Mirza.2016	III	2016	Niraparib vs Placebo	Experimental: niraparib (300 mg) qd Control: placebo	maintenance monotherapy	372/181	platinum-sensitive recurrent, high grade serous ovarian cancer	gBRCA mutation non gBRCA mutation	Experimental:21.0 months Control:5.5 months (HR:0.27, *P* < 0.0001)
Lauraine 2017	III	2017	Olaparib vs Placebo	Experimental: olaparib (300 mg) bid Control: placebo	maintenance monotherapy	196/99	platinum-sensitive relapsed ovarian cancer patients	BRCA1/2 mutation	Experimental:19.1 months Control:5.5 months (HR:0.30, *P* < 0.0001)
Coleman 2017	III	2017	Rucaparib vs Placebo	Experimental: rucaparib 600 mg bid Control: placebo	maintenance monotherapy	375/189	platinum-sensitive recurrent, high-grade ovarian carcinoma	BRCA1/2 mutation BRCA wild-type	Experimental:16·6 months Control:5.4 months (HR:0.23, *P* < 0.0001)
Moore 2018	III	2018	Olaparib vs Placebo	Experimental: olaparib (300 mg) bid Control: placebo	maintenance monotherapy	260/131	platinum-sensitive high grade serous or endometrioid ovarian, primary peritoneal, or fallopian tube carcinoma	BRCA1/2 mutation	Experimental:36 months longer Control:13.8 months (HR:0.30, *P* < 0.0001)
Coquard 2019	III	2019	Olaparib plus bevacizumab vs Bevacizumab	Experimental: olaparib (300 mg) bid plus bevacizumab Control: placebo plus bevacizumab	combination with bevacizumab for maintenance therapy	537/269	platinum status unknown high-grade serous or endometrioid ovarian cancer, primary peritoneal cancer, or fallopian-tube cancer	BRCA1/2 mutation BRCA wild-type BRCA status unknown	Experimental:37.2 months Control:21.7 months (HR:0.31, *P* (no data provided))
Martin 2019	III	2019	Niraparib vs placebo	Experimental: niraparib (200 mg) qd Control: placebo	maintenance monotherapy	487/246	platinum status unknown high-grade serous or endometrioid ovarian cancer, primary peritoneal cancer, or fallopian-tube cancer	BRCA mutation BRCA wild-type Non BRCA mutation	Experimental:22.1 months Control:10.9 months (HR:0.40, *P* < 0.001)
Coleman 2019	III	2019	Veliparib vs placebo	Experimental: veliparib (400 mg) bid Control: placebo	combination with chemotherapy and maintenance monotherapy	382/375	platinum status unknown high-grade serous epithelial ovarian, fallopian tube, or primary peritoneal carcinoma	BRCA mutation BRCA wild-type Non BRCA mutation	Experimental:34.7 months Control:22.0 months (HR:0.40, *P* < 0.001)

gBRCA mutation means the presence of a germline BRCA mutation; non gBRCA mutation means the absence of a germline BRCA mutation; bid means twice a day; qd means once daily.

### Overall survival (OS)

Oza 2014, Ledermann 2016, Lauraine 2017, Moore 2018 and Martin 2019 had assessed OS in ovarian cancer patients, while the maturity of OS analysis data in these four trials was 49%, 70%, 24%, 21% and 10.8% respectively, which means that the OS data were immature. By pooling the data from Oza 2014, Ledermann 2016, Lauraine 2017 and Moore 2018, OS in PARPis group seemed to have an advantage over placebo group in BRCA mutation setting (HR = 0.78, 95%CI = 0.61–1.01, fixed-effect model; *P* = 0.06, which did not meet the required threshold for statistical significance [*P* < 0.05]) (Figure 2A). The analysis data for the BRCA status unclassified group were extracted from Oza 2014, Ledermann 2016 and Martin 2019, and disappointingly there was no statistically significant beneficial effect for OS between the two groups (HR = 0.84, 95%CI = 0.61–1.15, *P* = 0.27, random effect model) (Figure 2B).

**Figure 2:** Pooled HRs of OS comparing PARPis maintenance therapy arm with Placebo maintenance therapy arm in ovarian cancer patients with BRCAm (**A**) and BRCA status unclassified (**B**)

### Progression-free Survival (PFS)

After pooling the data, it showed that there were 1319 patients with ovarian cancer with BRCA wild-type, including 750 in PARPis group and 569 in control groups, and PFS was significantly improved in the PARPis group than in the placebo group (HR = 0.53, 95%CI = 0.43–0.68, *P* < 0.00001, random effect model) (Figure 3A). Especially, data from all RCTs were pooled to analyze ovarian cancer patients with BRCA mutations, and when comparing the two groups (PARPis group, *n* = 1270; placebo group, *n* = 699), the median PFS HR was 0.30 (95%CI = 0.26–0.34, *P* < 0.00001, fixed-effect model) (Figure 3B). Six trials also analyzed the PFS of the BRCA status unclassified mainly consisting of BRCA mutation and BRCA wild-type, and the pooled HR of median PFS was 0.52 (95%CI = 0.41–0.66, *P* < 0.00001, random effect model) (Figure 3C). Significantly, three trials classified BRCA mutation status in more detail, and in patients with BRCA1m and with BRCA2m, the HRs of median PFS were 0.38, 0.23, respectively (95%CI = 0.29–0.48, *P* < 0.00001, fixed effect model; 95%CI = 0.10–0.57, *P* = 0.001, random effect model) (Figure 3D,E).

**Figure 3:** Pooled HRs of PFS comparing PARPis maintenance therapy arm with Placebo maintenance therapy arm in ovarian cancer patients with BRCAwt (**A**), BRCAm (**B**), BRCA status unclassified (**C**), BRCA1m (**D**) and BRCA2m (**E**)

### Adverse event (AEs)

Data of AEs extracted from selected literature were used to risk analysis, as details are shown in Table 2. In total, a treatment-emergent adverse event of any grade occurred in 2685 of 2725 patients (98.53%) who received PARPis and in 1495 of 1602 patients (93.32%) who received placebo (RR = 1.05, 95%CI = 1.03–1.07, *P* < 0.00001, fixed-effect model). Most notably, PARPis significantly increased the overall risk to suffer grade≥3 AEs and serious AEs compared with placebo (grade≥3 AEs: incidence rate = 55.19%, RR = 2.16, 95%CI = 1.47–3.18, *P* < 0.0001, random effect model; serious AEs: incidence rate = 26.29%, RR = 1.82, 95%CI = 1.32–2.51, *P* < 0.00001, random effect model). In PARPis group, for any grade events, the five most common AEs of any grade were nausea, fatigue, anaemia, vomiting and thrombocytopenia, and for grade ≥3 AEs, they were anaemia, thrombocytopenia, neutropenia, fatigue and nausea. Considering the incidence and relative risk of AEs, we found that hemotoxicity and gastrointestinal reactions may be the main obstacles to the clinical use of PARPis.

**Table 2:** Summary of treatment-emergent adverse events

Summary of adverse events						
Adverse events	Grade	PARPis (adverse events/ total patients) (%)	Placebo (adverse events/ total patients) (%)	RR	95%CI	*P* value (test for over effect)
Patients with any adverse event	Any	2685/2725 (98.53)	1495/1602(93.32)	1.05	1.03-1.07	<0.00001
	≥3	1504/2725(55.19)	427/1602(26.65)	2.16	1.47-3.18	<0.0001
Serious adverse events	–	635/2415(26.29)	201/1291(15.56)	1.82	1.32-2.51	<0.00001
Nausea	Any	1786/2725(65.54)	504/1602(31.46)	1.98	1.63-2.42	<0.00001
	≥3	71/2725(2.60)	11/1602(0.68)	3.60	1.99-6.53	<0.0001
Fatigue	Any	1414/2725(51.89)	556/1602(34.70)	1.39	1.23-1.57	<0.00001
	≥3	145/2725(5.32)	25/1602(1.56)	3.54	2.32-5.41	<0.00001
Anaemia	Any	1136/2725(41.68)	167/1602(10.42)	3.56	2.43-5.21	<0.00001
	≥3	537/2725(19.70)	18/1602(1.12)	13.01	4.90-34.54	<0.00001
Vomiting	Any	836/2725 (30.67)	226/1602(14.10)	2.19	1.92-2.51	<0.00001
	≥3	48/2725(1.76)	15/1602(0.93)	1.82	1.03-3.24	0.04
Thrombocytopenia	Any	715/2589(27.61)	58/1474(3.93)	5.60	3.29-9.54	<0.00001
	≥3	315/2589(12.16)	6/1474(0.40)	10.77	2.11-49.94	0.004
Constipation	Any	724/2725(26.56)	278/1602(17.35)	1.33	1.05-1.70	0.02
	≥3	10/2725(0.36)	4/1602(0.24)	1.11	0.39-3.17	0.85
Diarrhea	Any	658/2725(24.14)	339/1602(21.16)	1.16	0.99-1.35	0.06
	≥3	32/2725(1.17)	16/1602(0.99)	1.11	0.62-2.00	0.73
Abdominal pain	Any	623/2725(22.86)	386/1602(24.09)	0.94	0.81-1.09	0.40
	≥3	49/2725(1.79)	22/1602(1.37)	1.37	0.83-2.26	0.22
Neutropenia	Any	597/2725(21.90)	171/1602(10.67)	2.14	1.40-3.26	0.0004
	≥3	279/2725 (10.23)	65/1602 (4.05)	2.77	1.40-5.46	0.003
Headache	Any	556/2725(20.40)	218/1602(13.60)	1.48	1.13-1.93	0.004
	≥3	10/2725 (0.36)	8/1602(0.49)	0.70	0.31-1.59	0.40
Dysgeusia	Any	387/1931(20.04)	55/1047(5.25)	3.54	2.18-5.77	<0.00001
	≥3	1/1931(0.05)	0/1047 (0)	1.50	0.06-36.70	0.80
Decreased appetite	Any	492/2725(18.05)	160/1602(9.98)	1.79	1.51–2.21	<0.00001
	≥3	9/2725(0.33)	4/1602 (0.24)	1.18	0.41–3.40	0.76
Arthralgia	Any	491/2725(18.01)	308/1602 (19.22)	0.94	0.83–1.07	0.36
	≥3	11/2725(0.40)	5/1602(0.31)	1.11	0.45–2.72	0.82
Cough	Any	294/1880(15.63)	121/1024(11.81)	1.44	0.98–2.13	0.07
	≥3	1/1880(0.05)	1/1024(0.09)	0.51	0.05–4.87	0.56
Abdominal pain upper	Any	155/1029(15.06)	54/601(8.99)	1.69	1.26–2.26	0.0004
	≥3	2/1020(0.19)	1/601(0.16)	0.98	0.14–6.79	0.99
Dyspepsia	Any	206/1396(14.75)	70/780(8.97)	1.70	1.32–2.20	<0.0001
	≥3	1/1396(0.07)	0/780(0)	1.53	0.06–37.33	0.79
Dyspnoea	Any	312/2213(14.09)	76/1108(6.85)	2.05	1.62–2.61	<0.00001
	≥3	13/2213(0.58)	5/1108(0.45)	1.22	0.46–3.28	0.69
Dizziness	Any	360/2725(13.21)	134/1602(8.36)	1.58	1.31–1.92	<0.00001
	≥3	5/2725(0.18)	4/1602(0.24)	0.69	0.26–1.87	0.47
Hypomagnesaemia	Any	76/633(12.00)	35/343(10.20)	1.16	0.65–2.05	0.61
	≥3	1/633(1.57)	3/343(0.87)	0.33	0.05–2.03	0.23
Back pain	Any	305/2659(11.47)	154/1547(9.95)	1.15	0.96–1.38	0.13
	≥3	7/2659(0.26)	2/1547(0.12)	1.71	0.26–11.23	0.58
Nasopharyngitis	Any	87/764(11.38)	41/461(8.89)	1.31	0.91–1.86	0.14
	≥3	0/764(0)	0/461(0)	NE	NE	NA
Abdominal distension	Any	118/1359(8.68)	85/740(11.48)	0.76	0.59–0.99	0.04
	≥3	0/1359(0)	1/740(0.13)	0.16	0.01–3.98	0.27

## Discussion

Rapid progression or lower OS after cytoreductive surgery plus conventional cytotoxic chemotherapy for ovarian cancer patients indicates an urgent need for a new and effective treatment regimen. In addition to BRCA mutation related to the sensitivity of PARPis therapy, many studies have demonstrated that loss of DNA repair proteins of other tumor suppressor factors, many of which are related to homologous recombination deficiency, also induces such sensitivity to PARPis [29–32]. These studies suggested that the effectiveness of PARPis was mainly based on the defect of homologous recombination pathway, not only on the mutation of BRCA [29–32]. Through the results of clinical trials of PARPis in cancer patients and the growing understanding of various DNA repair defects, it was found that these drugs were effective for patients regardless of the mutation status of BRCA [33,34]. In ovarian cancer, these targeted inhibitors were the standard treatment for advanced serous ovarian cancer with BRCA mutation [35,36], and could also be used as alternative treatment for many patients other than BRCA germline mutation carriers [33,36].

At present, some scholars have analyzed the effect of PARPis on the treatment of ovarian cancer patients through meta-analysis [37,38]. However, more randomized controlled trials have been included in this study, including some of the latest clinical trials. What’s more, we analyzed the PFS and OS of ovarian cancer patients treated with PARPis more specifically, as well as the AEs related to PARPis in more detail. By integrating data from 9 RCTs, this meta-analysis discussed the efficacy and safety of various PARPis maintenance therapy including olaparib, niraparib,veliparib and rucaparib in the patients with ovarian cancer. Our research revealed an impressive efficacy of the PARPis maintenance therapy in treatment ovarian cancer patients with BRCAm or BRCAwt, in which the pooled HRs for PFS were 0.30 (95%CI = 0.26–0.34, *P* < 0.00001, fixed-effect model), and 0.53 (95%CI = 0.42–0.68, *P* < 0.00001, random effect model), respectively, comparing with placebo. The lifetime risk of ovarian cancer was different between BRCA1 and BRCA2 mutation carriers [3,39,40]. Consequently, their prognosis may be different. Bolton et al. [41] discovered that the 5-year overall survival of ovarian cancer was 44% for BRCA1 carriers and 52% for BRCA2 carriers. Similarly, Somlo et al. [42] confirmed that the clinical benefit and median PFS was a statistically higher for BRCA2 versus BRCA1 patients with metastatic breast cancer when treated with PARPi veliparib. Similarly, we confirmed that treating with PARPis, the clinical efficacy of patients with BRCA2m was better than that of patients with BRCA1m, with HRs for PFS being 0.23, 0.38 (BRCA2m: HR = 0.23, 95%CI = 0.10–0.57, *P* = 0.001, random effect model; BRCA1m: HR = 0.38, 95%CI = 0.29–0.48, *P* < 0.00001, fixed-effect model), respectively. A recent meta-analysis explored the impact of BRCA1 and BRCA2 mutations on survival of ovarian and breast cancer, and claimed that these mutations should be considered when designing appropriate treatment strategies [43]. Although many researchers believed that PARPis can be used to treat ovarian cancer without considering the BRCA status [33,36], the mutation status of BRCA provides a strong basis for the design of reasonable individualized targeted therapy for ovarian cancer. Therefore, to provide suitable treatment for ovarian cancer patients, it is suggested that ovarian cancer specimens after surgery need not only routine means for pathological examination, but also need gene testing to identify the relevant genotypes.

Earlier, Kaye et al. claimed that olaparib 400 mg twice per day was more suitable for patients because they found that 400 mg (8.8 months, 95% confidence interval = 5.4–9.2 months) was better than 200 mg (6.5 months, 95% confidence interval = 5.5–10.1 months) for median PFS time [44]. Thus, does the dosage of PARPis affect the prognosis of patients with ovarian cancer? Five groups of clinical trials involving olaparib maintenance therapy showed that compared with the control group, the hazard ratio of PFS ultimately obtained seemed to be positively correlated with the maintenance dose. Therefore, the appropriate treatment dose was also an aspect to be considered in the follow-up study. In addition, OS did not seem to differ significantly between patients treated with PARPi versus placebo, but the total number of patients was small and overall survival data was immature so that the study was not powered to make formal comparisons.

Our meta-analysis also provided an overview of the expected safety and tolerance of single-agent PARPi that could be of value to discuss treatment risk and benefit ratio with patients. PARPis have been gradually approved for clinical applications, so the evaluation of treatment-emergent AE is indispensable. AEs may lead to dosage adjustment, discontinuation of treatment, and even affect the health and safety of patients. A meta-analysis of 2479 patients treated with PARPis from 12 randomized controlled trials showed that incidences of severe neutropenia, thrombocytopenia, and anemia in patients receiving PARPis were 32.9%, 15.9% and 9.1%, respectively, which indicated that PARPis treatment increased the risk of severe hematologic toxicities [45]. Hematologic toxicities caused by PARPis are more common and serious, so it is necessary to monitor complete blood counts regularly. Because PARP inhibition is not selective to cancer cells, it eliminates the important mechanism of DNA repair of blood cells which are replaced more frequently like cancer cells, thus enhancing blood toxicity. In addition to increasing the risk of hematologic toxicities, another study showed that PARPis treatment significantly increased the risk of gastrointestinal toxicities at all levels in patients with ovarian cancer, except for constipation [46]. The frequent AEs recorded in these nine clinical trials that led to discontinuation of treatment and death in patients with PARPis were similar, which included anemia, thrombocytopenia, neutropenia, abdominal pain, intestinal obstruction, myelosuppression, nausea and vomiting. However, there are fewer cases of interruption of treatment and death due to AEs. Overall, PARPis seems to have a tolerance profile suitable for long-term maintenance therapy, but the high incidence rates for grade≥3 AEs and serious AEs are a trouble that cannot be ignored in clinical application.

## Abbreviations

95% CI: 95% confidence interval
AE: adverse event
HR: hazard ratio
NA: not applicable
NE: not estimable
OS: overall survival
PARP: poly ADP ribose polymerase
PFS: progression-free survival
RR: relative risk
